This article has been retracted.

# Effect of Dexmedetomidine on Cardiac Output among Parturient with Severe Preeclampsia after Cesarean Section

**DOI:** 10.1155/2022/4742350

**Published:** 2022-04-14

**Authors:** Yanxiang Lv, Ying Zhou, Yuan Qiao, Rui Hu, Yan Liang, Yanan Lian, Tongqiang He

**Affiliations:** Department of Obstetrics and Gynecology Intensive Care Unit, Northwest Women and Children's Hospital, Xi'an 710032, China

## Abstract

This study was to investigate the hemodynamic effect of dexmedetomidine among parturient with severe preeclampsia after cesarean section. Parturient with severe preeclampsia were randomly allocated to receive dexmedetomidine (0.2-0.7 *μ*g/kg/h) or equivalent volumes of 0.9% saline as control after cesarean section, respectively. A total of 36 parturient with severe preeclampsia were enrolled, including 18 in the dexmedetomidine (DEX) group and 18 in the saline group. Compared with the saline group, among those in the DEX group, CO was reduced by 1.30 L/min (95% CI: -2.36 to 0.25; *P* = 0.019). Additionally, HR (-13.79 bpm, 95% CI: -22.02 to -5.58; *P* = 0.002), SBP (-16.11 mmHg, 95% CI: -30.56 to -1.66; *P* = 0.030), DBP (-10.48 mmHg, 95% CI: -18.27 to -2.69; *P* = 0.002), and MAP (-12.36 mmHg, 95% CI: -22.05 to -2.66; *P* = 0.014) were reduced in the DEX group compared with the saline group. In contrast, there were no changes observed in SV and ICON between groups. In conclusion, dexmedetomidine reduces cardiac output by inhibiting the acceleration of heart rate without sacrificing myocardial contractility and stroke volume.

## 1. Introduction

Preeclampsia is the most common complication of pregnancy affects 2% to 8% of pregnancies [1, 2]. This disorder of pregnancy increases maternal and fetal morbidity as well as mortality prominently. Various complications [3–5], such as eclampsia, heart failure, and exacerbated or persistent hypertension, still occur frequently in parturient with preeclampsia postpartum, especially with pain, anxiety, and scare postoperative. Sedation and analgesia are widely recommended as an approach to control agitation, blunt the stress response, and reduce metabolism in intensive care unit (ICU) [6]. Timely sedation postpartum could minimize patient discomfort that may obtain many benefits. However, specific recommendations for patients with severe preeclampsia are lacking in postoperative sedation.

Dexmedetomidine, a highly selective *α*-2-receptor agonist, is a first-line sedative medication in ICU and has been increasingly used for obstetric anesthesia. Dexmedetomidine, which provides light sedation, possesses analgesic, sympatholytic, anxiolytic properties and attenuates the stress response without significant respiratory depression [7, 8]. Due to the short half-life, dexmedetomidine was undetectable in milk at 24 hours after discontinuation of the administration and conducive to the early conversion of infant feeding to exclusive breastfeeding [9], suggesting that dexmedetomidine is compatible with breastfeeding [10]. Theoretically, dexmedetomidine might make it an ideal sedative for parturient with severe preeclampsia postoperative. We designed this study to explore the hemodynamic security of dexmedetomidine in parturient with severe preeclampsia after cesarean section.

## 2. Methods

### 2.1. Inclusion Criteria and Exclusion Criteria

This prospective, randomized, and controlled study was approved by the Ethics Committee of Northwest Women and Children's Hospital (NWCH; approval number: 21-048). The inclusion criteria were patients with severe preeclampsia over 18 years old and patients who received cesarean section in the Department of Obstetrics and Gynecology Intensive Care Unit, NWCH, from 1 January to 31 December 2019. The exclusion criteria were cardiovascular disease, sick sinus syndrome or atrioventricular block, bradycardia (heart rate < 50 beats·min^−1^), multiple pregnancies, allergy to dexmedetomidine, currently receiving antipsychotic drugs, eclampsia, or acute heart failure before cesarean section.

### 2.2. Usual Management

All participants signed informed consent and were divided into two groups randomly using a computer-generated table of random numbers. Every patient equally received a usual postoperative care including administration of oxytocin, magnesium sulfate for seizure prophylaxis, analgesia, and antihypertensive agent. Antihypertensive medications were administrated when systolic blood pressure ≥ 160 mmHg and/or diastolic blood pressure ≥ 110 mmHg. All patients received analgesia protocol consisted of 100 *μ*g sufentanil diluted into 100 mL postoperative.

### 2.3. Interventions

In the DEX group, patients received continuous infusion of dexmedetomidine without loading dose at a rate of 0.2-0.7 *μ*g/kg/h to achieve RASS score in the target range on the night of surgery. The target of sedation scores on the Richmond Agitation and Sedation Scale was −2 to +1 (lightly sedated to restless), on which scores range from −5 [unresponsive] to +4 [combative], as assessed at least every 2 hours. The saline group received equivalent volumes of saline. If bradycardia occurred which was defined as heart rate < 50 beats·min^−1^, the infusion of dexmedetomidine was terminated and the patient was excluded from the study.

### 2.4. Diagnostic Criteria

Severe preeclampsia met the Clinical Management Guidelines for Obstetrician-Gynecologists of ACOG criteria for preeclampsia diagnosis and fulfilled one of the severe features [11]: systolic blood pressure ≥ 160 mmHg and/or diastolic blood pressure ≥ 110 mmHg; severe persistent right upper quadrant or epigastric pain not accounted for by alternative diagnoses and abnormally elevated liver enzymes which indicated impaired liver function; renal insufficiency; thrombocytopenia; pulmonary edema; new-onset headache; and visual symptom.

### 2.5. Outcome Measures

The primary outcome was the change of cardiac output (CO) from baseline. Secondary outcomes included the change of other hemodynamic variables from baseline: stroke volume (SV), index of contractility (ICON), heart rate (HR), systolic blood pressure (SBP), diastolic blood pressure (DBP), and mean arterial blood pressure (MAP). Variables were obtained before dexmedetomidine or saline administration as baseline and at 10 hours after dexmedetomidine or saline administration, respectively. Adverse events such as eclampsia, heart failure, bradycardia, and nausea and vomiting (PONV) were monitored and recorded. The hemodynamic variables were obtained by the ICON™ monitor, a noninvasive hemodynamic monitoring device (Osypka Medical, Berlin, Germany).

### 2.6. Statistical Analysis

Study data from Lee et al. showed a decrease of CO from 3.72 ± 1.0 L/min at baseline to 2.90 ± 0.5 L/min at 20 min after administration in the DEX group with no changes (from 3.61 ± 1.1 L/min to 3.87 ± 1.4 L/min) in the saline group. A two-sided 0.05 level of significance and a sample size of 36 patients (18 per group) provided 80% statistical power to demonstrate this difference in CO. To accommodate for a 10% attrition rate, we will recruit a total of 40 patients (PASS11, independent t tests; allocation ration = 1).

The normality of the data distribution was verified by the Shapiro-Wilk tests. For continuous data, means with standard deviations (SDs) were presented. The changes of hemodynamic variables were calculated as the value after drug administration minus the value at baseline. Mean differences were expressed with their 2-sided 95% confidence intervals. Independent-samples *t* tests were performed for between-group differences. Within-group comparisons from baseline to drug administration were tested with paired-samples *t* tests. All statistical analyses were conducted with SPSS 25.0 software package, a 2-sided *P* value of <0.05 was considered statistically significant.

## 3. Results

From the 64 patients who met the enrollment criteria, 40 patients agreed to participate. Thirty-six parturient with severe preeclampsia completed the study, 18 in each group, respectively (Figure 1).

Demographic characteristics and baseline of hemodynamic variables were similar in the two groups (Table 1).

As Figure 2 shows, CO decreased by 0.10 ± 0.68 L/min in the DEX group and significantly increased by 1.2 ± 1.7 L/min in the saline group compared with baseline. The change in CO was significantly different between groups by -1.30 L/min (95% CI: -2.36 to 0.25; *P* = 0.019). Similarly, HR was remarkably accelerated in the saline group and significantly reduced in the DEX group compared with the saline group (-13.79 bpm; 95% CI: -22.02 to -5.58; *P* = 0.002). No changes were observed in SV and ICON in either group (-7.63 mL, 95% CI: -17.83 to 2.57; *P* = 0.133), (-8.27, 95% CI: -21.22 to 4.69; *P* = 0.1.94).

Systolic blood pressure (-16.11 mmHg, 95% CI: -30.56 to -1.66; *P* = 0.030) and diastolic blood pressure (-10.48 mmHg, 95% CI: -18.27 to -2.69; *P* = 0.002) as well as mean arterial blood pressure (-12.36 mmHg, 95% CI: -22.05 to -2.66; *P* = 0.014) were also significantly reduced in the DEX group compared with the saline group (Figure 3).

Five patients in the DEX group received antihypertensive medication and 6 in the saline group during study period (27.8% vs. 33.3%, *P* > 0.05). No major adverse events such as eclampsia and heart failure were recorded during the study. Three patients reported nausea and vomiting in both groups after intervention.

## 4. Discussion

The most important finding of present study is the infusion of dexmedetomidine without loading dose reduce cardiac output by attenuated heart rate in patients with severe preeclampsia postoperative but does not impair stroke volume and index of contractility. It is also suggested that the administration of dexmedetomidine decrease blood pressure.

Several researches reported the effects of dexmedetomidine on cardiac function. Lee et al. [12] assessed cardiac function in healthy patients during general anesthesia by the echocardiographic examinations and found that dexmedetomidine did not impair biventricular systolic and diastolic function but decreased cardiac output by reducing heart rate. Snapir et al. [13] reported that dexmedetomidine significantly reduced CO and HR of healthy male subjects in parallel with a reduction in myocardial oxygen demand and did not induce evident myocardial ischemia but caused a decrease in SV when the dosage exceed the recommended therapeutic level. Additionally, escalading dose of dexmedetomidine also led reduced CO and SV [14, 15]. However, high dose effect of dexmedetomidine on CO is contrary in animal experiment [16]. A series of animal experiments [17–21] showed that dexmedetomidine prevents myocardial dysfunction via multiple signaling pathways. A meta-analysis [22] showed that dexmedetomidine is an efficacious cardioprotective drug in adults and children undergoing cardiac surgery. Compared to previous studies, the present study was conducted in women with preeclampsia. Preeclampsia is a pathological condition, which is accompanied with reduced compensatory function associated with hypertension and myocardial ischemia. In consideration of loading dose transient hypertension reported [23], we adopted a method of continuous infusion at recommended rate without loading dose [2] in patients with severe preeclampsia postoperative. Our study reveals that dexmedetomidine reduces cardiac output by inhibiting the acceleration of heart rate without sacrificing myocardial contractility and stroke volume. According to these data, we can infer that patients with severe preeclampsia may benefit from dexmedetomidine by decelerating heart rate and therefore reducing cardiac work and myocardial oxygen consumption.

Previous studies have reported that administration of dexmedetomidine provided a significant hemodynamic stability during cesarean section in patients with preeclampsia [24–28]. There is very little published research on administration of dexmedetomidine for postoperative sedation of preeclampsia patients. A few of the published studies showed that dexmedetomidine sedation in eclampsia patients were effective in reducing blood pressure [29–31]. This also accords with our research, which showed that blood pressure was significantly reduced after dexmedetomidine administration. However, all of these studies did not evaluate the effects of dexmedetomidine on cardiac function. We monitored the effects of dexmedetomidine on cardiac function in patients with severe preeclampsia by noninvasive hemodynamics technology for the first time. It is the strength of this study.

## 5. Limitations

The first limitation is associated with lack of blinding. The unblinded manner may have introduced subjective bias by clinicians. In addition, the plasma concentration of dexmedetomidine was not measured, which may be useful to determine whether plasma concentration varied hemodynamic effects, especially on cardiac function. Thirdly, we did not monitor the plasma level of cortisol and noradrenaline, which could improve our understanding in the potential mechanism of dexmedetomidine on hemodynamic.

## 6. Conclusion

In conclusion, dexmedetomidine may reduce the risk of heart failure by reducing cardiac work and cardiac afterload. Sedation should be routinely performed in parturient with severe preeclampsia after cesarean section to cope with adverse events caused by stress, pain, postoperative hypertension, and increased cardiovascular volume.

## Figures and Tables

**Figure 1:** Flow diagram of the studied patients enrolled in the study.

**Figure 2:** Changes in cardiac output. (a) Change from baseline to the end of treatment in cardiac output; (b) change from baseline to the end of treatment in stroke volume; (c) change from baseline to the end of treatment in index of contractility; (d) change from baseline to the end of treatment in heart rate. DEX: dexmedetomidine; CO: cardiac output; SV: stroke volume; ICON: index of contractility; HR: heart rate; CI: confidence interval.

**Figure 3:** Changes in blood pressure. (a) Change from baseline to the end of treatment in systolic blood pressure; (b) change from baseline to the end of treatment in diastolic blood pressure; (c) change from baseline to the end of treatment in mean arterial blood pressure. DEX: dexmedetomidine; SBP: systolic blood pressure; DBP: diastolic blood pressure; MAP: mean arterial blood pressure; CI: confidence interval.

**Table 1:** Baseline demographic and clinical characteristics (mean ± SD).

	DEX (*n* = 18)	Saline (*n* = 18)	*P*
Age (year)	30.50 ± 4.82	32.22 ± 4.13	0.259
BMI (kg/m^2^)	29.03 ± 2.95	28.61 ± 3.05	0.675
Delivery week	34.90 ± 2.23	35.02 ± 2.66	0.878
CO (L/min)	4.66 ± 0.88	4.46 ± 1.15	0.560
HR (bmp)	82.94 ± 12.16	78.00 ± 11.93	0.227
SV (mL)	56.11 ± 8.08	57.28 ± 10.40	0.709
ICON	37.92 ± 7.92	38.76 ± 12.06	0.806
SBP (mmHg)	143.67 ± 11.75	138.56 ± 13.19	0.228
DBP (mmHg)	94.56 ± 9.40	92.56 ± 9.62	0.532
MAP (mmHg)	110.22 ± 9.16	107.83 ± 10.29	0.467

DEX: dexmedetomidine; BMI: Body Mass Index; CO: cardiac output; HR: heart rate; SV: stroke volume; ICON: index of contractility; SBP: systolic blood pressure; DBP: diastolic blood pressure; MAP: mean arterial blood pressure.

## Data Availability

The data used to support the findings of this study are available from the corresponding author upon request.
